The article "LncRNA FBXL19-AS1 promotes breast cancer cells proliferation and invasion via acting as a molecular sponge to miR-718" was retracted in 2023. Reasons: duplicated images; signs of a paper mill; concerns about the data.

# LncRNA FBXL19-AS1 promotes breast cancer cells proliferation and invasion via acting as a molecular sponge to miR-718

**DOI:** 10.1042/BSR20182018

**Published:** 2019-04-02

**Authors:** Zhenmin Ding, Pengcheng Ye, Xiaohu Yang, Hongmiao Cai

**Affiliations:** Department of Anesthesia, Shanghai East Hospital, Tongji University School of Medicine, Shanghai 200120, China

**Keywords:** breast cancer, lncRNA FBXL19-AS1, miR-718

## Abstract

Long non-coding RNAs (lncRNAs) have been suggested to serve vital roles in tumor initiation and progression. However, the expression and underlying mechanisms of lncRNA FBXL19-AS1 in breast cancer (BC) remain unclear. In the present study, we found that FBXL19-AS1 expression was significantly up-regulated and correlated with advanced clinical features and poor overall survival of BC patients. Functionally, FBXL19-AS1 inhibition suppressed BC cells proliferation, invasion, and epithelial–mesenchymal transition (EMT) processes *in vitro* and reduced tumor growth *in vivo*. In addition, we found that FBXL19-AS1 might function as a ceRNA to sponge miR-718, and miR-718 could rescue the effects of FBXL19-AS1 on BC cells progression. Therefore, these findings suggested that FBXL19-AS1 might serve as an oncogenic lncRNA and promoted BC progression by sponging miR-718, indicating FBXL19-AS1 could serve as a potential therapeutic target for BC treatment.

## Introduction

Breast cancer (BC) is one of the most commonly occurring female malignant tumors, with an increased incidence and much younger onset age recently [1,2]. Despite noteworthy advances in screening, surgery, and chemo-radiotherapy techniques, the prognosis of BC patients remains unsatisfactory [3,4]. Therefore, it was of great significance to investigate the mechanisms underlying BC progression.

Long non-coding RNA (lncRNA) is a group of non-coding RNA transcripts with more than 200 nucleotides in length, and lacking the protein translation abilities [5,6]. Accumulating evidence reported that lncRNAs play critical roles in various cellular processes, such as cell growth, apoptosis, metastasis, and differentiation [7,8]. For example, Zhang et al. [9] revealed that MALAT1 up-regulation correlated with clear cell renal cell carcinoma progression and poor prognosis. Guo et al. [10] revealed that SNHG20 could function as an oncogenic lncRNA by regulating miR-140-5p-ADAM10 axis and MEK/ERK signaling pathway in cervical cancer. Gao et al. [11] found that HOTAIR facilitated leukemogenesis by enhancing self-renewal of leukemia stem cells through epigenetic silencing of p15. However, the roles and underlying mechanism of lncRNAs in tumor progression remain unclear.

In the present study, we explored the expression, biological functions, and underlying mechanisms of FBXL19-AS1 in BC progression. Our data showed that FBXL19-AS1 could promote BC progression by acting as a molecular sponge to modulate miR-718 expression.

## Materials and methods

### Clinical samples

A total of 49 pairs of BC tissues and their paired adjacent normal tissues (ANT) were obtained from patients receiving surgery at Shanghai East Hospital from 2015 to 2017. Their BC conditions were diagnosed by two pathologists following the American Society of Clinical Oncology guidelines [12]. The obtained upon resection tissue samples were immediately snap-frozen in liquid nitrogen and then stored at −80 °C until further use. All patients in this study signed the informed consent. This study was approved by the Research Scientific Ethics Committee of Shanghai East Hospital.

### Cell culture and transfection

Human BC cell lines (MDA-MB-231, ZR-75-1, MCF-7, BT-549, MDA-MB-468, and T47D) and the normal mammary fibroblast cell line (Hs578Bst) were purchased from Cell Bank of Chinese Academy of Sciences (Shanghai, China). All cell lines were cultured in DMEM (Gibco, Carlsbad, CA, U.S.A.) supplemented with 10% fetal bovine serum (FBS, Gibco) at 37°C in 5% CO_2_.

To down-regulate FBXL19-AS1 expression in BC cells, small interference RNA targeting FBXL19-AS1 (si-FBXL19-AS1) and scrambled negative control (si-NC) were designed and synthesized by GenePharma (Shanghai, China). MiR-718 mimics, miR-718 inhibitors, and corresponding negative controls were purchased from RiboBio (Guangzhou, China). Lipofectamine 2000 reagents (Invitrogen, Carlsbad, CA, U.S.A.) were used to perform all transfection with the instruction of manufacturer’s protocol. The sequences of si-FBXL19-AS1 were as follows: si-RNA-1, 5′-CAAGGTACACGGTAGCGTAGCTTA-3′; si-RNA-2, 5′-GAGUGUAATGCATUUAGUTT-3′.

### RNA extraction and quantitative RT-PCR

Total RNA from tissues and cells were extracted with TRIzol reagent (Invitrogen) according to the manufacturer’s protocol. cDNA was synthesized from total RNA by a PrimerScript RT Reagent kit (Takara, Japan). MiRNA from total RNA was reverse transcribed using the Prime-Script miRNA cDNA Synthesis Kit (Takara). Then qRT-PCR was performed with the SYBR green Premix Ex Taq II (Takara) in an ABI 7900HT system (Applied Biosystems, Foster City, CA, U.S.A.). GAPDH and U6 were used as internal controls for mRNA and miRNA, respectively. The relative gene expression was calculated using the 2^−∆∆C^_t_ method. The primers were as follows: FBXL19-AS1 sense, 5′-GGTACAACTACGGATATGA-30, and reverse, 5′-TACGTCTCGACCATTACGCA-3′.

### Cell Counting Kit (CCK)-8 assay

Cell Counting Kit-8 (CCK-8; Dojindo, Japan) was used to measure the proliferation of cancer cells. The transfected cells (5 × 10^4^ cells/well) were seeded in 96-well plates and incubated for 24, 48, 72, and 96 h. CCK-8 reagents were added to each well, and then incubated for another 4 h. The absorbance at 450 nm was measured using a Microplate Reader (Bio‐Rad, Hercules, CA, U.S.A.).

### Colony formation assay

Transfected cells at a density of 1 × 10^3^ cells/well were plated into 6-well plates and maintained in DMEM medium. Medium was replaced every 3 days. After 2 weeks, colonies were fixed with methanol, and then stained with 0.1% crystal violet. Colonies with over 50 cells were manually counted.

### Cell invasion assay

Transwell chambers (8 μm pores, Corning, NY, U.S.A.) were used for invasion evaluation. Briefly, the transwell chambers were pre-coated with Matrigel (BD, San Jose, CA, U.S.A.). Cells were seeded in the upper chamber, and medium with 10% FBS was added in the lower chamber. After 24 h, the cells not invaded were removed by a cotton swab. Invaded cells were fixed in 4% paraformaldehyde and stained by 0.1% crystal violet for 15 min. The number of cells on the membrane was counted under a microscope (Nikon, Japan).

### Xenograft assay

Four-week-old athymic male BALB/c nude mice were randomly assigned to two groups. MCF7 cells (2 × 10^6^) transfected with sh-FBXL19-AS1 and sh-NC were subcutaneously injected into the right flank of nude mice (Cancer Institute of the Chinese Academy of Medical Science). The Institutional Animal Ethics Committee of Shanghai East Hospital approved this animal study. The size of tumor was measured every 7 days. Seven weeks after inoculation, mice were killed and tumors were isolated. Tumor volume was calculated as the following formula: (length × width^2^)/2.

### Dual luciferase reporter assay

The FBXL19-AS1 fragment containing the miR-718 binding site was amplified by PCR and cloned into the psiCHECK-2 vector (Promega, Madison, WI, U.S.A.). The QuickChange^®^ Site-Directed Mutagenesis Kit was used to mutate the binding site of FBXL19-AS1. Cells were co-transfected with luciferase reporter vectors comprising FBXL19-AS1-Wt or FBXL19-AS1-Mut and miR-718 mimics using Lipofectamine 2000 (Invitrogen). The firefly and Renilla luciferase activity was measured 48 h post-transfection using the dual-luciferase reporter assay system (Promega).

### RIP assay

RIP assay was performed by using Magna RNA-binding protein immunoprecipitation kit (Millipore, Billerica, MA, U.S.A.). The cells were collected and lysed using RIP lysis buffer containing protease inhibitor and RNase inhibitor. Whole-cell extracts were incubated with RIP buffer containing magnetic beads conjugated with anti-Ago2 antibody for 1 h. Following digesting protein with proteinase K, the immunoprecipitated RNA was extracted for qRT-PCR analysis.

### Western blot

Cells were lysed with ice-cold RIPA buffer containing protease inhibitor (Roche, Mannheim, Germany). The concentrations were measured using BCA protein assay kit (Pierce, Rockford, IL, U.S.A.). Proteins were separated using 10% SDS–PAGE and transferred to polyvinylidene difluoride membranes (PVDF, Millipore). Following blocking with a 5% skim milk solution, membranes were incubated at 4°C overnight with specific antibodies against E-cadherin, N-cadherin, and GAPDH (Abcam, Cambridge, U.K.). Subsequently, the membranes were incubated with HRP-conjugated secondary antibody (Cell Signaling, Danvers, MA, U.S.A.) at room temperature for 1 h. The final data were detected with ECL detection system (Millipore).

### Statistical analysis

All experimental data were presented as means ± standard deviation (SD) of three independent experiments and processed by SPSS 20.0 software (IBM, Armonk, NY, U.S.A.). Students *t* test and one‐way analysis of variance (ANOVA) were used to explore the significant difference of groups. *P*<0.05 was considered to be statistically significant.

## Results

### FBXL19-AS1 was up-regulated in BC

Firstly, we determined FBXL19-AS1 expression in 49 pairs of BC tissues. QRT-PCR showed that FBXL19-AS1 expression was significantly up-regulated in BC tissues compared with ANT (Figure 1A; *P*<0.05). Interestingly, high FBXL19-AS1 expression was associated with BC patients with lymphnode metastasis (LM) and advanced TNM stage (II + III) (Figure 1B,C; *P*<0.05). GEPIA database further confirmed that FBXL19-AS1 expression was significantly up-regulated in BC tissues (Figure 1D,E; *P*<0.05). In addition, qRT-PCR showed that FBXL19-AS1 expression was increased in BC cell lines (MDA-MB-231, ZR-75-1, MCF-7, BT-549, MDA-MB-468, Bcap37, and T47D) compared with Hs578Bst cells (Figure 1F; *P*<0.05).

**Figure 1:** FBXL19-AS1 was up-regulated in BC (**A**) QRT-PCR was used to explore FBXL19-AS1 expression in BC tissues and ANT. (**B**) FBXL19-AS1 expression was increased in BC patients with LM compared with patients with NLM. (**C**) FBXL19-AS1 expression was up-regulated in BC patients with TNM stage II + III compared with TNM stage I. (**D**) FBXL19-AS1 expression in BC was analyzed by using GEPIA database. (**E**) FBXL19-AS1 was slightly up-regulated at stages I–IV and X using GEPIA database. (**F**) QRT-PCR was used to explore FBXL19-AS1 expression in BC cell lines and normal mammary fibroblast cells. ^*^P<0.05. Abbreviation: NLM, none lymphnode metastasis.

### FBXL19-AS1 promoted BC cells proliferation, invasion, and EMT processes *in vitro*

To explore the roles of FBXL19-AS1 in BC tumorigenesis, MDA-MB-231 and MCF-7 cells were transfected with si-FBXL19-AS1 and si-NC (Figure 2A; *P*<0.05). CCK-8 assay and colony formation assay showed that FBXL19-AS1 inhibition significantly reduced BC cells proliferation and colony formation abilities (Figure 2B,C; *P*<0.05). Transwell assay revealed that FBXL19-AS1 suppression significantly reduced BC cells invasion abilities (Figure 2D; *P*<0.05). The epithelial–mesenchymal transition (EMT) has been recognized as a key regulator of metastasis of BC. Therefore, we explored whether FBXL19-AS1 regulated EMT process in BC cells. Results showed that FBXL19-AS1 inhibition significantly induced the expression of epithelial marker E-cadherin and decreased mesenchymal marker N-cadherin both in mRNA and protein levels (Figure 2E,F; *P*<0.05). These results indicated that FBXL19-AS1 might play critical roles in BC progression.

**Figure 2:** FBXL19-AS1 promoted BC cells proliferation and invasion (**A**) Relative expression of FBXL19-AS1 in BC cells transfected with si-FBXL19-AS1 or si-NC. (**B**,**C**) CCK-8 assay and colony formation assay were used to measure BC cells viability. (**D**) Transwell invasion assay was used to explore BC cells invasion ability. (**D**) QRT-PCR was used to determine E-cadherin and N-cadherin mRNA levels in BC cells. (**E**) Western blot was used to measure E-cadherin and N-cadherin protein levels in BC cells. *P<0.05.

### FBXL19-AS1 negatively regulated miR-718 expression in BC

Recently, studies showed that lncRNAs could act as a competing endogenous RNA (ceRNA) or a molecular sponge to interact with miRNAs and participate the physiological and pathological processes [13]. Using the online software program DIANA, miR-718 was found to potentially bind to FBXL19-AS1 (Figure 3A). Dual-luciferase reporter assay showed that miR-718 mimics significantly reduced the luciferase activity of FBXL19-AS1-Wt in BC cells (Figure 3B; *P*<0.05). QRT-PCR showed that FBXL19-AS1 knockdown remarkably increased miR-718 expression in BC cells (Figure 3C; *P*<0.05). Moreover, RIP assay showed that FBXL19-AS1 and miR-718 were co-immunoprecipitated by the anti-Ago2 antibody (Figure 3D; *P*<0.05). In addition, we showed that miR-718 expression was significantly decreased in BC tissues and cell lines (Figure 3E,F; *P*<0.05). Correlation analysis revealed that FBXL19-AS1 expression was negatively correlated with miR-718 expression in BC tissues (Figure 3G; *P*<0.05). Those data indicated that FBXL19-AS1 might act as a molecular sponge for miR-718 in BC cells.

**Figure 3:** FBXL19-AS1 acted as a sponge of miR-718 (**A**) The predicted miR-718 binding sites in FBXL19-AS1. (**B**) Dual luciferase reporter assay showed that miR-718 mimics significantly decreased the luciferase activity of FBXL19-AS1-Wt in BC cells. (**C**) FBXL19-AS1 inhibition increased miR-718 expression in BC cells. (**D**) RIP assay showed that miR-718 and FBXL19-AS1 were both enriched in Ago2-containing miRNAs. (**E**,**F**) QRT-PCR was used to explore miR-718 expression in BC tissues and cell lines. (**G**) FBXL19-AS1 expression was negatively correlated with miR-718 expression in BC tissues. *P<0.05.

### MiR-718 rescued the effects of FBXL19-AS1 on BC tumorigenesis

Next, we transfected si-FBXL19-AS, miR-718 inhibitors (anti-miR-718), or anti-miR-718 + si-FBXL19-AS into MCF-7 cells. CCK-8 assay and colony formation assay showed that miR-718 inhibitors promoted MCF-7 cells proliferation and colony formation abilities, and miR-718 inhibitors could reverse the effects of FBXL19-AS1 knockdown on BC cells (Figure 4A,B; *P*<0.05). Transwell invasion assay indicated that miR-718 inhibitors increased MCF-7 cells invasion ability, and miR-718 inhibitors could abolish the effects of FBXL19-AS1 knockdown on BC cells (Figure 4C; *P*<0.05). Thus, these data suggested that miR-718 might act as a tumor suppressor in BC progression, and miR-718 could rescue the effects of FBXL19-AS1 on BC tumorigenesis.

**Figure 4:** The effects of FBXL19-AS1 were mediated by regulating miR‐718 (**A**,**B**) CCK-8 and colony formation assays were used to determine cells viability of BC cells transfected with anti-miR-718, si-FBXL19-AS1, and anti-miR-718 + si-FBXL19-AS1. (**C**) Transwell invasion assay was used to explore BC cells invasion ability. (**D**,**E**) Suppression of tumor growth was observed by FBXL19-AS1 inhibition. (**F**) Immunohistochemistry of Ki-67 in xenograft tumor tissues. (**G**) FBXL19-AS1 and miR-718 expression in xenograft tumor tissues were examined by qRT-PCR. *P<0.05

### FBXL19-AS1 promoted tumor growth *in vivo*

To further explore the oncogenic roles of FBXL19-AS1 *in vivo*, a xenograft tumor model was established. Results showed that FBXL19-AS1 knockdown significantly reduced tumor growth *in vivo* (Figure 4D,E; *P*<0.05). Ki-67 staining showed that FBXL19-AS1 inhibition decreased the Ki-67 positive staining cells compared with sh-NC group (Figure 4F; *P*<0.05). Moreover, qRT-PCR showed that the expression of miR-718 was increased and FBXL19-AS1 was decreased in xenograft tumors (Figure 4G; *P*<0.05). Therefore, we indicated that FBXL19-AS1 could promote BC tumorigenesis *in vivo*.

## Discussion

LncRNAs may originate from different regions of the genome, including the antisense strand or the introns of protein-coding genes, the promoters or untranslated regions of protein-coding genes, or even as independent transcripts within and outside of protein-coding genes [14]. Increasing evidence implicated that lncRNAs are vital to the development and prognosis of BC [15]. For example, Zhang et al. [16] showed that lncRNA CCAT1 was up-regulated and associated with poor overall survival and progression-free survival of BC patients. Zou et al. [17] found that MALAT1 promoted proliferation and invasion via targeting miR-129-5p in triple-negative BC. Luan et al. [18] found that lncRNA MIAT promoted BC progression and functioned as ceRNA to regulate DUSP7 expression by sponging miR-155-5p. However, the roles and underlying mechanisms of lncRNA in BC remain unclear.

Recently, FBXL19-AS1 has been reported to play a carcinogenic role in human cancers and is related to tumor metastasis. For example, Shen et al. [19] showed that lncRNA FBXL19-AS1 could play oncogenic role in colorectal cancer by sponging miR-203. Pan et al. [20] suggested that lncRNA FBXL19-AS1 regulated osteosarcoma cell proliferation, migration, and invasion by sponging miR-346. However, the functions and underlying mechanisms of FBXL19-AS1 in BC remain unclear. In the present study, we showed that FBXL19-AS1 expression was up-regulated and associated with advanced TNM stage, lymph node metastasis, and poor overall survival of BC patients. Function assays revealed that FBXL19-AS1 suppression reduced BC cell proliferation, invasion *in vitro* and reduced tumor growth *in vivo*. These results suggested that FBXL19-AS1 might act as an oncogenic lncRNA in BC progression.

MiRNAs are short non-coding RNA molecules with 20–24 nucleotides, and play important roles in the post-transcriptional regulation of gene expression [21]. Recently, increasing studies showed that lncRNAs act as ‘sponges’ to bind with specific miRNAs and then regulate multiple diseases [22]. For example, Zhang et al. [23] revealed that lncRNA HNF1A-AS1 promoted cell proliferation and invasion via regulating miR-17-5p in non-small-cell lung cancer. Chen et al. [24] revealed that lncRNA CCAT1 promoted multiple myeloma progression by acting as a molecular sponge of miR-181a-5p to modulate HOXA1 expression. In the present study, we identified miR-718 as a direct target of FBXL19-AS1. Luciferase report and RIP assays showed that FBXL19-AS1 could bind to miR-718 in BC cells. Previous studies showed that miR-718 could play important roles in tumor progression. For example, Wang et al. [25] found that miR-718 inhibited papillary thyroid cancer cell proliferation, metastasis, and glucose metabolism by negatively regulating the Akt-mTOR signaling pathway. Schrauder et al. [26] revealed that miR-718 was significantly decreased in BC. However, the function and underlying mechanism of miR-718 in BC remain unclear. In the present study, we found that miR-718 was significantly decreased and inversely associated with FBXL19-AS1 expression in BC tissues. Function assays showed miR-718 reduced BC cells viability and invasion; moreover, miR-718 inhibitors could abolish the effects of FBXL19-AS1 knockdown on BC cells. Thus, these findings indicated that FBXL19-AS1 exerted its oncogenic roles in BC at least in part by regulating miR-718 expression.

In conclusion, we demonstrated that lncRNA FBXL19-AS1 is highly expressed in BC, and promote the proliferative and invasive potentials of BC cells by functioning as a molecular sponge of miR-718. FBXL19-AS1 might serve as a potential therapeutic target for BC treatment.

## Abbreviations

ANT: adjacent normal tissue
BC: breast cancer
CCK: Cell Counting Kit
ceRNA: competing endogenous RNA
EMT: epithelial–mesenchymal transition
FBS: fetal bovine serum
si-FBXL19-AS1: small interference RNA targeting FBXL19-AS1
si-NC: scrambled negative control
